This article has been retracted.

# Prediction and Analysis of Autism Spectrum Disorder Using Machine Learning Techniques

**DOI:** 10.1155/2023/4853800

**Published:** 2023-07-10

**Authors:** Muhammad Shuaib Qureshi, Muhammad Bilal Qureshi, Junaid Asghar, Fatima Alam, Ayman Aljarbouh

**Affiliations:** ^1^Department of Computer Science, School of Arts and Sciences, University of Central Asia, Naryn, Kyrgyzstan; ^2^Department of Computer Science & IT, University of Lakki Marwat, KPK 28420, Pakistan; ^3^Gomal Centre of Pharmaceutical Sciences, Faculty of Pharmacy, Gomal University Dera Ismail Khan, KPK, Pakistan; ^4^Department of Computer Science, Shaheed Zulfikar Ali Bhutto Institute of Science and Technology, Islamabad 44000, Pakistan

## Abstract

Autism spectrum disorder is a severe, life-prolonged neurodevelopmental disease typified by disabilities that are chronic or limited in the development of socio-communication skills, thinking abilities, activities, and behavior. In children aged two to three years, the symptoms of autism are more evident and easier to recognize. The major part of the existing literature on autism spectrum disorder is covered by a prediction system based on traditional machine learning algorithms such as support vector machine, random forest, multiple layer perceptron, naive Bayes, convolution neural network, and deep neural network. The proposed models are validated by using performance measurement parameters such as accuracy, precision, and recall. In this research, autism spectrum disorder prediction has been investigated and compared using common parameters such as application type, simulation method, comparison methodology, and input data. The key purpose of this study is to give a centralized framework to use for researchers working on autism spectrum disorder prediction. The best results were obtained by using the random forest algorithm as it performs better than other traditional machine learning algorithms. The achieved accuracy is 89.23%. The workflow representations of the investigated frameworks assist readers in comprehending the fundamental workings and architectures of these frameworks.

## 1. Introduction

Due to its diverse genetic structure and compound neural connectivity, the human brain is the most structured and complex body organ. A scale-free network is called a neuronal connection between neurons, as it changes with enhancement. The more knowledge the brain receives, the more synaptic associations are formed, and then the analysis becomes more complicated. The connection between cognitive growth and functional brain wiring improves the interpretation of neurological disorder [1]. Owing to the irregular wiring between the various brain areas, autism is one of the heterogeneous and psychological growth disorders [2]. A neurodevelopmental disorder is known as the autism spectrum disorder (ASD) [1] that affects communication and behavior. The rise in the number of people suffering from ASD worldwide demonstrates a significant need for the implementation of ASD prediction models that are efficient and easy to execute. The nature of these models differs greatly with time and skill, and to understand this diversity, the idea of an autism spectrum has been implemented [3]. Around 50% of autistic children suffer from mental impairment. Some have aberrantly enlarged brain size, one-third have had at least two late adolescent epileptic seizures, and around half have a significant speech impairment [4]. Some autistic children have analytical abilities that are highly developed and this originated the word *autism spectrum disorder*. The ASD comprises of an autism disorder, Asperger's syndrome, and pervasive developmental disorder, not otherwise mentioned [5]. Genetic factors play a significant role in ASD. Autism is convincingly attributed to genetic mutations, gene deletions, variations of copy number (CNVs), and other genetic anomalies [6].

Some individuals with ASD are very verbal and communicative, while others do not use any means of communication that are verbal. Additionally, some individuals with ASD are very distracted from all aspects of social contact, while others have relationships and careers [7]. Studies show that the brain development of ASD individuals grows differently from the brain of typical controls. Autism is the most rapid developmental disorder in male and is four times more common than in female [8].

In fact, the ASD identification depends mainly on the medical experience used during direct interviews to determine patient's behavior [9]. The last 25 years are of great importance because it has seen enormous improvements in the detection of autism at an early stage. Before children learned vocabulary and iconic play skills, there was a debate about whether they could recognize autism. Improvements in early activity and structural changes in the brain have been reported in 6–12 month-old babies who continue to develop autism [10]. Machine learning algorithms can be used to evaluate data and obtain the finest biological markers from hundred biological markers if they have sufficient amount of data and also have high computation power [11]. The authors in [12] have used deep neural networks (DNNs) to classify ASD in functional magnetic resonance imaging (fMRI), recognizing the analytical decision-making driven by data and predict ASD.

The motivation behind this study is to present a method for diagnosing the autism spectrum disorder with the help of a better and accurate machine learning model. In order to predict the autism spectrum disorder, the machine learning algorithm provides an exact answer to the medical treatment system.

The major contributions of this research work are as follows:

- Balanced and scale data technique is used to test whether it affects the performance?
- Feature selection technique is applied to select optimal features from the whole dataset for prediction,
- Better machine learning-based autism spectrum disorder prediction model is proposed that predicts autism with better accuracy and improves the performance.

## 2. Previous Studies on Autism Spectrum Disorder Prediction

This section explains previous studies that use machine learning-based approaches to detect and predict the autism spectrum disorder. The main motive is to analyze and find some limitations to propose a new, better, and improved machine-learning based approach for autism spectrum disorder prediction.

Table 1 describes some acronyms that are used in this paper.

Automated algorithms for disease detection are being deeply studied for usage in healthcare. Graph theory and machine learning algorithms were used. For each age range being examined, the pipeline automatically selected 10 biomarkers. In discriminating between ASD and HC, measures of centrality are the most operational [11]. The study [13] used a neural network-based feature selection method from teacher-student which was suggested to have the most discriminating features and applied different classification algorithms. The results are compared with the already presented methods at the overall and site level. The authors in [14] also utilize the neural network to acquire the distributions of PCD for the classification of ASD as it has far more hyper parameters that make the model extra versatile. Payabvash et al. [15] used computer leaning algorithms to classify children with autism based on tissue connectivity metrics, hence, observed decreased connectome edge density in the longitudinal white matter tracts. It illustrated the viability of it in identifying children with ASD, connectome-based machine-learning algorithms. Emerson et al. [16] shows how functional neuroimaging can reliably predict which individuals obtain a clinical diagnosis of ASD at 24 months with 6-month-old infants at high familial risk for ASD.

In ref [17], the authors simulated machine learning techniques on data acquired from rest-state brain imaging to diagnose autism. The drawback of the proposed research is that it does not use any best feature selection method with repeating periods of 2s (sites NYU, SDSU, UM, USM). This led to a dataset of 147 ASD subjects and 146 balanced controls. The authors in [18, 19] conclude that the data may be used to establish diagnostic biomarkers for the progression of autism spectrum disorders and to distinguish those with the condition in the general population. Wang et al. [20] proposed an ASD identification approach which focuses on multi-atlas deep feature representation and ensemble learning technique. In study [21], the multimodal automated disease classification system uses two types of activation maps to predict whether the person is healthy or has autism. It was able to achieve 74% accuracy. Rakić et al. [22] suggested a technique which is based on a system composed of autoencoders and multilayer perceptron. Because of a multimodal approach that included a set of structural and functional data classification classifiers, the highest classification precision was 85.06%. In study [23], advanced deep-learning algorithms are proposed where HPC solutions can increase the accuracy and time of broad fMRI data analysis significantly. The authors in [24] explain what the results of machine learning studies may mean for the ultimate objective of determining an ASD biomarker that is uniquely sensitive and precise. However, the results cannot be applied to the entire ASD functional continuum. The study did not include evidence from other developmental conditions and was thus unable to specifically assess the specificity of typical CRF connections. Thomas et al. [25] introduced a novel analysis technique to identify changes in population dynamics in functional networks under ASD. They have also introduced machine learning algorithms to predict the class of patients with ASD and normal controls by using only population trend quality metrics as functions. The limitation of this approach is that the outcomes of the classification are highly dependent on the threshold parameter *T.* Another problem is that despite age variations in the experimental samples, the same spatial normalization design was used for all subjects. The authors in ref [26] proposed a collection of new features based on MRI images using machine learning algorithms to diagnose ASD which achieved 77.7% accuracy using the LDA approach.

Yin et al. [27] developed deep learning methods from functional brain networks built with brain functional magnetic resonance imaging (fMRI) data for the diagnosis of ASD. Another study [28] used a graph-based classification approach which yields better results but missing values are not handled and data normalization is not applied. A previous study [29] analyzes and works on brain networks which are inherent. It is deduced that ASD may be caused due to the aberrant mechanisms. The underlying individual variations in ASD symptom severity may be dysfunction in SN and visual systems and associated processes. Smith et al. [30] suggest that a weakened interaction with RSN temporal entitlement (RSN) and a higher degree of symptom severity in ASD people is correlated with the association with symptoms of the autism spectrum disorder. The findings suggest that FC and entropy provide additional details on the temporal spatio-organization of the brain. The authors in [31] proposed a novel element-wise layer incorporating general prior convictions built for connectomes and utilizes Brain-Net CNN and L2 regularization algorithm for classification purposes. The technique was validated using the K-Fold cross-validation method. However, this study does not utilize any pre-processing and feature selection technique as it highly affects the accuracy of the model. A multichannel deep attention neural network called DANN was proposed in [32] in which mechanism-based learning with attention achieved a precision of 0.732. However, this study is limited because the selected cohort is in the population of teenagers and young adults, and hence, restricting the generalizability of the model since the diagnosis of ASD was carried out much earlier. Alvarez‐Jimenez et al. [33] presented a multiscale descriptor to classify brain regions and recognize those with discrepancies between groups using a 2D representation and the curvelet transform. With regards to the state-of-the-art methods, including those focused on deep learning, it is shown to be successful. Another study [34] used the scope of the brain network's Laplacian matrix and topology centrality as characteristics. This study utilizes the features that are presented in [26] and acquired 79.2% accuracy. The study [35] suggested a novel architecture using CNN which has to identify autism and monitor patients using RS-fMRI data. This study concludes that through structural MRI images, 3D convolutionary neural networks can also be used to distinguish healthy subjects and patients with autism. Sherkatghanad et al. [36] suggested a CNN architecture. The mean accuracy of the presented model which used 234 test data is 70.2% but no feature selection technique was utilized. The authors in [19] indicate that deep learning techniques can classify broad multi-site datasets accurately which may be useful for the potential application of machine learning to identify psychological conditions. The authors in [37] suggest the ANN algorithm for multisite data and also shares the importance of network connectivity for classification was linked to verbal communication deficits in autism. The study [38] utilizes deep neural network and atlases for classification and acquired the accuracy of 78.07% on real data and 79.13% on augmented data.

## 3. Proposed Model

The proposed model presented in Figure 1 is a concept of a system made up of the composition of ideas that are used by optimal feature selection to help people learn, understand, or estimate the prediction of autism spectrum disorder. The main purpose of the conceptual model is to communicate the basic principles and characteristics of the system reflected by it. The computational model is built to offer an interpreted understanding of the framework to the consumers of the software.

The proposed model consists of six major steps that are as follows: (1) data collection as data are collected from ABIDE and ABIDE collected data using 17 different sites, (2) data pre-processing which includes following steps such as if missing values present then they are imputed rather than deletion, the whole dataset scaled at same scale to improve results, the number of instances in dataset for two classes has been balanced, outliers first detected than removed from dataset for its biasness in results, and features have been selected using machine learning technique, (3) data splitting technique which splits data into testing, training, and validation datasets, (4) classification model uses four different classifiers such as SVM, MLP, NB, and RF to check which classifier performs the best with selected dataset, (5) model evaluation is performed using parameters like accuracy, precision, and recall, and (6) validation is carried out using the k-fold mechanism.

## 4. Materials and Methods

### 4.1. Experimental Setup

In Google Co Labs, a free online cloud-based Jupyter Notebook environment is used. Python packages are used for pandas for loading the data set; NumPy for handling the subsets, and pilots for making plots. The pre-processing includes making subsets, selection of best features, removal of missing values, and the application of SMOTE is performed using the programming language Python in the Jupyter Notebook. The machine learning steps are also implemented in Python. To put the features in a better format and split the data in the test and train NumPy was used. To cross-validate the model, sklearn library was used. To smoothly run and validate the proposed model, machine having specification of Windows 10, CPU 2.9 GHz core i7, GPU Intel HD Graphics 620, RAM 12 GB, and free disk space of minimum 5 GB was used for experiments.

### 4.2. Data

The dataset used in this study is retrieved from the widely recognized ABIDE dataset used by many researchers [11, 13, 14, 16–36]. The dataset aims to diagnose whether or not a patient has autism based on certain diagnostic measures in the dataset. The collection of such instances from a broader database was subject to certain restrictions. In particular, all patients are males aged between 7 and 64 years. The datasets consist of multiple variables of medical predictors and one objective variable, the outcome. Predictor variables include the size of the functional voxel, age, etc. The ABIDE dataset consists of the 1112 subjects' rs-fMRI images, structural MRI images (T1-weighted), and phenotypic information. 539 of these are ASD while 573 are TC subjects as represented in Figure 2. Because of the diversity of the subjects, the ABIDE dataset is a very challenging dataset to work with instances.

### 4.3. Pre-Processing

#### 4.3.1. Missing Value Imputation

The number of missing values, however, is high. This step involves a data exploratory process to identify and handle the outliers by using the box plot approach. There were various missing values in the dataset, so the missing values were handled by an iterative imputer. In general, the data input method is better because it makes it possible to use as many samples for machine learning as possible. Iterative imputation is a method where every feature is shaped as a function of the other features, e.g., a regression problem where missing values are predicted. After missing value imputation, all of the features have 1112 instances and all missing values are vanished by using the iterative missing value imputation method.

#### 4.3.2. Outliers Detection

Outliers have been detected using box plot and then the interquartile range is defined which uses an upper limit and lower limit of column and removes the values which lie outside the limit. All the outliers are removed using this technique.

#### 4.3.3. SMOTE for Balancing the Dataset

The simplest methodology to cope with the imbalanced datasets is to oversample the minority class with replicating examples in the autism class. The SMOTE is the method that produces artificial instances on a random basis of the minority class from the nearest neighbors of the line joining the minority class sample to increase the number of the already available original instances. Therefore, these artificial instances are created on the basis of the original dataset features so that they become like the original instances of the minority class.

#### 4.3.4. Feature Selection with Sequential Forward Selection

Sequential forward selection (SFS) is used for feature selection due to its immense significance. We have used it because the used dataset is based on 1112 instances and 74 features which mean high dimensional which needs to exclude some features.

#### 4.3.5. Dataset Splitting

In this phase, total number of the autism patient dataset is split into two partitions for training and testing. With respect to the proposed model, training partition contained 70% data while remaining 30% data used for testing purpose. Literature describes 70-30 split strategy of input data. Out of total 1146 instances, 803 training instances were used for building classifying models of machine learning algorithms and remaining 343 training instances for testing partition were used to evaluate the built models.

### 4.4. Classification

We have used random forest with other machine learning techniques such as naive Bayes, support vector machine, and multiple layer perceptron algorithms.

#### 4.4.1. Random Forest (RF)

RF is a machine learning technique for solving classification and regression problems using decision tree algorithms. To train the 'forest' formed by the random forest method, a bagging or bootstrap aggregation method is used. To overcome the drawbacks of a decision tree algorithm, the random forest method is used. It decreases dataset overfitting and enhances accuracy. It makes predictions without requiring extensive package parameters (such as scikit-learn). Let ${\hat{c}}_{b}\left(x\right)$ be the class prediction of the *b*-th random-forest tree, then

(1) $$\begin{array}{c} {\hat{C}}_{xf}^{B}\left(x\right)={\left\{{\hat{C}}_{b}\left(x\right)\right\}}_{1}^{B}. \end{array}$$

#### 4.4.2. Naïve Bayes (NB)

The naive Bayes technique is a supervised learning procedure for tackling classification issues which is based on the Bayes theorem that makes predictions based on an object's probability. Bayes' theorem is numerically presented as follows:

(2) $$\begin{array}{c} P\left(A\;|\;B\right)=\frac{P\left(B\;|\;A\right)P\left(A\right)}{P\left(B\right)}, \end{array}$$

where *P*(*A|*/*B*) is the probability of hypothesis A on the observed event B which is known as posterior probability, *P*(*B|A*) is the probability of the evidence given that the probability of a hypothesis is true known as likelihood probability. *P*(*A*) is the probability of hypothesis before observing the evidence known as prior probability. *P*(*B*) is the probability of evidence known as marginal probability.

#### 4.4.3. Support Vector Machine (SVM)

SVM is a supervised classification technique that uses a line to distinguish between two separate groups. In many circumstances, the separation is not that straightforward. The hyperplane dimension must be altered from one to the *N*^th^ dimension in this scenario called as Kernel. To put it another way, it is the functional link that exists between the two observations.

#### 4.4.4. Multiple Layer Perceptron (MLP)

A family of functions is defined by an MLP or multilayer neural network. MLP is a type of feedforward artificial neural network (ANN). MLP, especially those with a single hidden layer, is commonly referred to as “vanilla” neural networks. There are at least three levels of nodes in an MLP: an input layer, a hidden layer, and an output layer. Each node with the exception of the input nodes is a neuron with a nonlinear activation function. Backpropagation is a supervised learning technique used by MLP.

### 4.5. Model Validation

Cross-validation is a mathematical method for assessing master learning abilities. The K-fold validation method is employed for validation. In the K-fold approach, the entire dataset serves as both training and testing. In this way, the entire dataset is tested by using 70% data for training and 30% data for testing against the test case and the findings are validated against the dataset.

### 4.6. Measurement

In this study, we used accuracy, recall, and precision for performance measurement as represented in (3)–(5).

(3) $$\begin{array}{c} \text{Precision}=\frac{\text{True Positive}}{\text{True Positive}+\text{False Positive}}, \end{array}$$

(4) $$\begin{array}{c} \text{Accuracy}=\frac{\text{True Negative}+\text{True Positive}}{\text{True Negative}+\text{True Positive}+\text{False Negative}+\text{False Positive}}, \end{array}$$

and

(5) $$\begin{array}{c} \text{Recall}=\frac{\text{True Positive}}{\text{True Positive}+\text{False Negative}}. \end{array}$$

Here, the term true positive indicates that the model predicts positive class correctly and true negative indicates that model predicts negative class correctly. The four classifiers RF, NB, MLP, and SVM are compared in Figure 3 on the basis of accuracy, precision, and recall.

## 5. Results and Discussion

The prediction of autism spectrum disorder was carried out on the basis of a traditional machine learning technique consisting SVM, NB, RF, and MLP. The techniques were applied on a dataset balanced by using SMOTE. The technique was applied on the 1146 instances of 16 features on balance dataset. The results were obtained after 50 iterations. The empirical performance of traditional machine learning algorithm-based classifiers is demonstrated in Table 2. According to the table, RF shows notable performance with respect to an accuracy of 94.73%. On the other hand, NB and MLP show better performance than SVM with respect to an accuracy of 91.86%, whereas SVM shows the least classification accuracy of 90.43%.

The RF gives a notable empirical result of 81.88% and 89.23% accuracy for imbalanced and balanced dataset, respectively. The NB gives 79.12% accuracy with imbalanced dataset; however, it gives 85.43% accuracy with balanced and scaled dataset. On the other hand, MLP gives 75.11% accuracy with imbalanced dataset and 81.84% with balanced dataset. Likewise, SVM gives 83.33% accuracy with imbalanced dataset but 80.43% with balanced dataset. It clearly shows that all traditional algorithms give improved accuracy with balanced and scaled dataset. The traditional four classifiers RF, NB, MLP, and SVM are compared on the basis of precision in Table 3.

It is clear that precision of RF with balanced dataset is 90.12% which is high as compared to the imbalanced data which is 82.56%. The NB gives precision of 77.23% and 84.52% with imbalance and balanced dataset. The MLP gives precision of 75.15% and 80.21% with imbalanced and balanced dataset. The SVM gives precision of 79.54% and 81.89% with imbalanced and balanced dataset, respectively. The four classifiers are compared in Table 4 on the basis of recall.

It is clear that recall of RF with balanced dataset is 88.33% which is high as compared to the recall with imbalanced data which is 80.58%. The NB gives recall of 78.32% and 81.43% with imbalanced and balanced dataset. The MLP gives recall of 72.23% and 77.58% with the imbalanced and balanced dataset. The SVM gives a recall of 75.65% and 80.55% with the imbalanced and balanced dataset, respectively.

## 6. Comparisons of Applied Classifier Techniques

We have implemented four classifiers RF, NB, MLP, and SVM algorithms where RF presents notable accuracy and precision performance as compared to the other traditional classifiers portrayed in Figures 4 and 5. Recall comparison is portrayed in Figure 6.

Table 5 shows accuracy comparison of the proposed autism prediction model with and without SMOTE.

## 7. Conclusion

The prediction model for the autism spectrum disorder plays a vital role in predicting autism and helps in diagnosing in time. In this research, we have surveyed prediction models for the autism spectrum disorder including different machine learning techniques. Theoretically, the working of these techniques have been evaluated and illustrated so that a new researcher can get started on a single board. The detailed comparison based on common parameters allows for the quick identification of architectural and implementation-related similarities and differences among various prediction models. We have given in-depth analysis which sets this study apart from other autism spectrum disorder techniques. Only autism spectrum disorder prediction techniques were consolidated in this study. The state-of-the-art ASD prediction using various machine learning techniques are comprehensively covered in this research but there are still plenty of opportunities for upcoming investigators.

As this model is better than state-of-the-art methods, but in future it can be tested with fuzzy logic algorithms for checking more accuracy for the autism spectrum disorder. In addition, other datasets can be experimented for a comparison purpose.

## Figures and Tables

**Figure 1:** ML-based ASD classification model.

**Figure 2:** Dataset before and after SMOTE. (a) Dataset before SMOTE. (b) Dataset after SMOTE.

**Figure 3:** Comparison of RF, NB, MLP, and SVM. (a) Accuracy. (b) Precision. (c) Recall.

**Figure 4:** Accuracies comparison in the line chart.

**Figure 5:** Precision comparison in the line chart.

**Figure 6:** Recall comparison in the line chart.

**Table 1:** Description of acronyms.

Acronym	Description
ASD	Autism spectrum disorder
DNN	Deep neural network
LDA	Linear discriminant analysis
SVM	Support vector machine
ANN	Artificial neural network
CDC	Centers for disease control and prevention
KNN	K-nearest neighbor
LR	Logistic regression
SMOTE	Synthetic minority over sampling technique
RF	Random forest
MLP	Multilayer perceptron
NB	Naïve Bayes
fMRI	Functional magnetic resonance imaging
FC	Functional connectome
RSN	Randomized subspace Newton

**Table 2:** Accuracy comparison of RF, NB, MLP, and SVM.

Traditional classifier	Accuracy (%)	
	Imbalanced dataset	Balanced dataset (SMOTE)
RF	81.88	89.23
NB	79.12	85.43
MLP	75.11	81.84
SVM	83.33	80.43

**Table 3:** Precision comparison of RF, NB, MLP, and SVM.

Traditional classifier	Precision (%)	
	Imbalanced dataset	Balanced dataset (SMOTE)
RF	82.56	90.12
NB	77.23	84.52
MLP	75.15	80.21
SVM	79.54	81.89

**Table 4:** Recall comparison of classifiers.

Traditional classifier	Recall (%)	
	Imbalanced dataset	Balanced dataset (SMOTE)
RF	80.58	88.33
NB	78.32	81.43
MLP	72.23	77.58
SVM	75.65	80.55

**Table 5:** Comparison of existing techniques and the proposed technique.

Ref/Year	Model	Accuracy (%)
[32] 2020	Multichannel DANN model with RF	65.9
[32] 2020	Multichannel DANN model with SVM	69.3
[22] 2020	Classification method using MLP	85.06
[15] 2018	Potential biomarker identification model based on NB	66
Proposed model		
	RF without balancing the dataset	81.88
	RF with balancing the dataset	89.23

## Data Availability

The dataset used in this study is retrieved from the widely recognized ABIDE (Autism Brain Imaging Data Exchange) dataset.
